# Analysis of the Effect of Intelligent Red Blood Cell Distribution Diagnosis Model on the Diagnosis and Treatment of Gastrointestinal Bleeding

**DOI:** 10.1155/2021/5216979

**Published:** 2021-11-12

**Authors:** Xibin Sun, Yuhong Zhang, Jiaxin Li, Bin Zhang, Qian Jia

**Affiliations:** ^1^The First Affiliated Hospital of Hebei North University, Department of Laboratory Medicine, Hebei, Zhangjiakou 07500, China; ^2^The First Affiliated Hospital of Hebei North University, Department of Obstetrics and Gynecology, Hebei, Zhangjiakou 07500, China

## Abstract

In order to explore the role of red blood cell distribution width in the diagnosis and treatment of gastrointestinal bleeding, this paper applies map feature recognition technology to red blood cell distribution broadband and constructs an intelligent red blood cell distribution width diagnosis model. To extract the content-level features of the image safely and effectively, this paper introduces the mechanism of jitter quantization to extract the content-level features at the lowest frequency of the image. In addition, this article employs an experimental approach to investigate the function of red blood cell distribution width in the diagnosis and management of gastrointestinal bleeding in the elderly. Finally, this article establishes an experimental group and a control group and then performs a research study using real-life hospital case studies. According to the statistical findings, the red blood cell distribution width index may play a significant role in the diagnosis and management of gastrointestinal bleeding, particularly in the case of severe bleeding.

## 1. Introduction

Red blood cell distribution width (RDW) is a parameter used to measure the width of red blood cell variables in a standard complete blood count report. In short, it is an objective indicator that reflects the unequal size of red blood cells. Compared with the observation of the red blood cell morphology and size on the blood smear, the red blood cell distribution width is more objective and accurate [1]. Generally, the standard volume of red blood cells is approximately in the range of 6–8 um. However, if some variations are encountered, the red blood cell volume variables will be significantly affected. The higher the red blood cell distribution width value, the larger the volume variable [2].

Current research shows that high levels of red blood cell distribution width values are considered to be caused by chronic inflammation and malnutrition. For this reason, the red blood cell distribution width is generally considered to be a marker of inflammation [3]. In various inflammation-related diseases, such as sepsis, acute coronary syndrome, and stroke, the distribution of red blood cells has potential diagnostic or prognostic significance. The breadth of red blood cell dispersion has slowly been a study topic in recent years. In patients with heart failure, coronary artery disease, or peripheral atherosclerosis, as well as healthy individuals, it may be utilised as an independent predictive risk factor for cardiovascular or cerebrovascular events. Moreover, it can also be used to assess cardiovascular risk factors in patients with rheumatoid arthritis. At the same time, it is closely related to the mortality of patients with sepsis and septic shock and has a certain predictive value. In digestive system diseases, the red blood cell distribution width has also become an effective diagnostic indicator.

Gastrointestinal bleeding is a more frequent critical emergency among patients in hospitals. According to the bleeding site, it can be divided into upper gastrointestinal bleeding and lower gastrointestinal bleeding. Upper gastrointestinal bleeding refers to the bleeding caused by lesions of the esophagus, stomach, duodenum, biliary tract, pancreas, and other organs above the Treitz ligament [4].

Clinically, gastrointestinal bleeding is usually divided into chronic bleeding and acute bleeding according to blood loss and speed. In patients with massive gastrointestinal bleeding and acute peripheral circulatory failure in a short period of time, the mortality rate is 3.6%–21%, and it is as high as 40.0% in the elderly and high-risk groups. There are many causes of gastrointestinal bleeding, and they are relatively complex. The severity and location of bleeding vary. It is critical to promptly and correctly identify the bleeding location and establish the treatment strategy. Upper gastrointestinal bleeding is the most frequent among them at the moment, with an annual incidence of approximately 150/100,000 and a fatality rate of 6 to 10%. If physicians are unable to identify and treat them immediately, patients' lives may be jeopardised.

The current research results on the causes, diagnosis, and treatment of upper gastrointestinal bleeding at home and abroad are as follows: the main common causes of upper gastrointestinal bleeding are peptic ulcer, acute gastric mucosal lesions, ruptured esophageal and gastric varices, and gastric cancer. Acute upper gastrointestinal bleeding in different age groups has a high incidence of peptic ulcer. Upper gastrointestinal bleeding requires different treatment options according to the degree of bleeding, the cause, and the amount of bleeding: conservative treatment is suitable for patients with chronic, small bleeding or gastrointestinal bleeding and unstable blood pressure, pulse, and respiration. This treatment can stabilize the vital signs of patients as soon as possible. Endoscopic hemostasis therapy is suitable for the following: patients with stable vital signs of gastrointestinal bleeding are the first choice. Esophageal and gastric varices bleeding is good, and it should be carried out within 24–48 hours after admission. Interventional therapy is suitable for patients with gastrointestinal bleeding whose site is difficult to identify by gastroscopy, large bleeding volume, and large amount of blood in the stomach. Surgery is suitable for patients with active hemorrhage who are not allowed to do other examinations or check the bleeding site, patients with persisting bleeding, patients with other diseases in the abdominal cavity, or patients whose medical and other treatment programs are ineffective.

Based on the above analysis, this paper applies the red blood cell distribution width to the diagnosis and treatment of gastrointestinal bleeding and combines computer intelligence technology to construct an intelligent diagnosis model to improve the diagnosis of gastrointestinal bleeding and reduce the adverse effects of gastrointestinal bleeding on patients.

## 2. Related Work

Gastrointestinal bleeding is a more frequent critical emergency among patients currently in the hospital. According to the bleeding site, it can be divided into upper gastrointestinal bleeding and lower gastrointestinal bleeding [5]. Clinically, gastrointestinal bleeding is usually divided into chronic bleeding and acute bleeding according to blood loss and blood loss speed [6]. Patients with massive gastrointestinal bleeding in a short period of time with acute peripheral circulatory failure have a mortality rate as high as 10% [7], and the mortality rate is as high as 40.0% in the elderly and high-risk groups [8]. There are many causes of gastrointestinal bleeding, which are relatively complicated, and the degree and location of bleeding are different. Therefore, clarifying the bleeding site and determining the treatment plan must be fast and accurate [9]. Moreover, it is very important to understand and pay attention to gastrointestinal bleeding. If clinicians cannot diagnose and treat them promptly and quickly, they may even endanger the life of the patient.

One of the main causes of peptic ulcers is *Helicobacter pylori* infection, and fewer patients are routinely tested for *Helicobacter pylori*. Although individuals are becoming increasingly worried about their health, most persons afflicted with *Helicobacter pylori* are unaware that they have been infected and have close contact with others, which contributes to *Helicobacter pylori* cross infection. At the same time, patients who know that they are infected with *Helicobacter pylori* fail to eradicate HP in time and infect the surrounding people, which is the main reason for the high incidence of the disease. The secondary cause of gastrointestinal bleeding is bleeding from esophageal and gastric varices [10]. At present, the incidence of chronic viral hepatitis B is high in my country and the world. It progresses to cirrhosis, and there is a greater risk of esophageal and gastric varices in decompensated cirrhosis. Moreover, the number of patients with alcoholic liver cirrhosis is increasing year by year, and this reason is the main cause of liver cirrhosis abroad. In addition, there are still drug users in the world, so patients with chronic hepatitis C are also on the rise, and the number of patients with liver cirrhosis is further increasing. According to the above reasons, the rupture and bleeding of esophageal and gastric fundus varices have become the second most important cause of acute upper gastrointestinal bleeding. Secondly, acute gastric mucosal lesions are the third cause. Acute gastric mucosal lesions may be caused by one of two things. One is drug-induced damage to stomach mucosal epithelial cells [11]. Nonsteroidal anti-inflammatory medications, such as aspirin and Celexa, are common. In recent years, the number of people suffering from hypertension and coronary heart disease in my country has been increasing year by year. As aspirin is the first choice for secondary prevention drugs, more patients take this drug for a long time, so the possibility of acute gastric mucosal lesions is increasing year by year. Another reason is alcoholism. The ethanol in alcohol can damage the lipoprotein layer on the gastric mucosa. At present, the number of people with alcoholism caused by heavy drinking for various reasons has increased significantly in recent years, and the risk of acute gastric mucosal lesions is higher than before [12].

Patients with acute gastrointestinal hemorrhage are required to stay in bed, do water fasting, keep the airway unobstructed, and open fluid passages when they are hospitalized. At the same time, they need to be monitored by ECG and closely monitor their consciousness, heart rate, blood pressure, respiration, body temperature, and other basic vital signs. In addition, patients with circulatory failure and shock should be given indwelling gastric tube and urinary catheter [13]. At the same time, it is necessary to monitor the patient's blood routine, liver and kidney function, and electrolyte changes every 2–4 hours and pay attention to whether there are blood transfusion indications, liver function damage, renal function damage, and electrolyte disorders. If the above symptoms are present, timely symptomatic treatment should be given [14]. In addition, all patients with acute gastrointestinal bleeding should complete their blood typing when they are admitted to the hospital to prepare for subsequent blood transfusion treatment in advance. At the same time, patients need to actively supplement blood volume to improve peripheral circulation [15]. To prevent multiple organ failures caused by microcirculation disorders, if necessary, symptomatic treatment of suspended red blood cells and plasma can be given. Therefore, the primary measures for acute gastrointestinal bleeding are antishock, rapid blood volume replacement, and stabilization of vital signs.

## 3. Red Blood Cell Distribution Width Diagnosis Algorithm

To extract the content-level features of the image safely and effectively, a jitter quantization mechanism is introduced to extract the content-level features at the lowest frequency of the image. Using the logistic mapping as in formula (1), a pseudorandom matrix is generated, and *λ* is the parameter value. This matrix is transformed into an integer matrix with only two elements of 1 and −1 [16]:

(1) $$\begin{array}{c} x_{n+1}=\lambda x_{n}\left(1-x_{n}\right). \end{array}$$

Among them, the initial value *x*_0_ can be used as a key. The sequence is converted into a jitter matrix *M*^*d*^.

The jitter matrix *M*^*d*^ is adjusted by the jitter factor *β* to change the jitter amplitude. Then, the adjusted dither matrix is added to the quantization matrix *M*^*q*^ to obtain the dither quantization matrix *Q*^*d*^:

(2) $$\begin{array}{c} Q^{d}=M^{q}\left(1+\beta \cdot M^{d}\right). \end{array}$$

The realization process of the jitter quantization matrix is shown in Figure 1.

For the low-frequency wavelet coefficient *L*, the jitter quantization matrix is used for quantization to obtain the quantized wavelet coefficient matrix *E* [17]:

(3) $$\begin{array}{c} E_{0}=\text{round}\left(\frac{LL_{2}}{Q^{d}}\right)\cdot Q^{d}. \end{array}$$

Figure 2 shows the specific implementation process of extracting content-level features.

The wavelet coefficient value grows closer and closer to 0 as the frequency increases, making it more sensitive to noise. This paper adopts the method of extracting energy features in the wavelet domain to quantize each frequency domain coefficient using the jitter quantization matrix *Q*^*d*^ and calculate the energy of each level of wavelet domain as the feature of constructing the hash:

(4) $$\begin{array}{c} E_{2}\left(i,j\right)=x_{HL2}^{2}\left(i,j\right)+x_{LH2}^{2}\left(i,j\right)+x_{HH2}^{2}\left(i,j\right),\\ E_{1}\left(i,j\right)=x_{HL1}^{2}\left(i,j\right)+x_{LH1}^{2}\left(i,j\right)+x_{HH1}^{2}\left(i,j\right). \end{array}$$

In the above formula, *E*_2_ is a robust level feature, and *E*_1_ is a detailed level feature.

The specific implementation process diagram is shown in Figure 3 [18].

In order to improve the robustness of the constructed perceptual hash, this paper uses the three-mean and quartile standard deviation of the generated feature matrix as the final feature [19].

The characteristic matrix coefficient sequence *x*_1_, *x*_2_,…, *x*_*n*_ is arranged from small to large and denoted as *x*_(1)_, *x*_(2)_,…, *x*_(*n*)_. The formula for calculating the median is

(5) $$\begin{array}{c} M=\left\{\begin{array}{cc} X_{\left(\left(n+1\right)/2\right)}, & n=1,3,5,\ldots ,\\ \frac{1}{2}\left(x_{\left(n/2\right)}+x_{\left(\left(n/2\right)+1\right)}\right), & n=2,4,6,\ldots . \end{array}\right) \end{array}$$

The median is a numerical feature that describes the location of the data center. Moreover, a significant feature of the median is that it is not easily affected by outliers and has strong robustness.

For 0 ≤ *p* ≤ 1 and *n* elements, its *p*-quantile is

(6) $$\begin{array}{c} M_{p}=\left\{\begin{array}{cc} X_{\left[np\right]+1}, & np=\notin Z,\\ \frac{1}{2}\left(X_{\left[np\right]+1}\right), & np\in Z. \end{array}\right) \end{array}$$

Among them, *Z* represents the set of integers, and [*np*] represents the integer part of np. When *p* = 0.75 and *p* = 0.25, they are called upper and lower quartiles, respectively.

The calculation formula for the three-mean value is

(7) $$\begin{array}{c} \hat{M}=\frac{1}{4}M_{0.25}+\frac{1}{2}M+\frac{1}{4}M_{0.75}. \end{array}$$

The three-mean value $\hat{M}$ is used to binarize the extracted multiple features to generate the final feature.

After extracting the features, chaotic cat mapping is used to scramble the coefficient coordinates of the feature matrix. The feature matrix is an *N* ^*∗*^*N* two-dimensional matrix, the coordinates of the elements are represented by (*i*, *j*), the coordinates of the elements after scrambling are represented by (*i*′, *j*′), and the cat mapping matrix is

(8) $$\begin{array}{c} A=\left[\begin{array}{cc} 1 & a\\ b & ab+1 \end{array}\right],\\ \left[\begin{array}{c} i^{\prime }\\ j^{\prime } \end{array}\right]=A\left[\begin{array}{c} i\\ j \end{array}\right]\left(\mathrm{mod}N\right). \end{array}$$

Among them, *a* > 0, *b* > 0 are natural numbers, generally *a* < *N*, *b* < *N*, and the parameters *a* and *b* are used as the key for the feature matrix scrambling. For the key of the scrambled cat mapping, we can introduce a method of mapping the key to a string and setting a meaningful password string to generate the key. The method of mapping ASCII code is used here, the ASCII code of the key string is taken, and they are converted to decimals for chaotic logistic mapping. After dozens of iterations, the key is obtained by operations such as linear expansion, modulo, and rounding.

The feature matrix scrambling has two consequences. One is to make hash extraction more secure. The extraction position of the hash is altered after the coefficients of the feature matrix are jumbled, making it more difficult for the attacker to reconstruct the hash. The second goal is to make the authentication hash more resistant to malicious assaults. The extraction of the hash in the feature coefficient matrix after scrambling is not focused on a specific section of the feature matrix but instead strengthens the connection between the hash and the entire feature matrix. Moreover, any modification of malicious attacks will affect the hash value extracted from the entire frequency domain level.

For the security of the scrambled keys *a*, *b*, considering the situation where the key is obtained by multiple mapping transformations, the calculation formula of the key space can be written:

(9) $$\begin{array}{c} K={\left(N-1\right)}^{2q}. \end{array}$$

Among them, N is the size of the feature matrix, and *q* > 0 is the number of mappings. It can be seen that the key space is related to the size of the square matrix and the number of times of mapping. The more the times of mapping, the more secure the key.

After feature extraction, two compressed feature schemes can be used to generate perceptual hash.

### 3.1. Scheme 1

The MD5 algorithm is used to hash each feature. From the hash codes generated by each feature, several bits are respectively extracted to combine to form an authentication hash code.

In order to make the hash extracted from the image have strong relevance and robustness to the image content and have the necessary properties for accurate hashing such as unidirectionality and collision resistance, the design idea of “robust feature plus accurate hash” is adopted. Robust feature extraction may remove superfluous information that is unrelated to the picture's content, integrate related data, decrease the amount of image data to a manageable level, and improve the relevance and robustness of the authentication hash and the image content. After the robust feature is extracted, the feature is accurately hashed so that the certified hash has all the characteristics of the accurate hash. This robust feature plus accurate hash mode can better balance the contradiction between the robustness and fragility of the authentication hash [20].

### 3.2. Scheme 2

The statistical method is used for compression, and each feature matrix is divided into data blocks with a size of 20 × 20. *M* represents the number of blocks the feature matrix is divided into. *N*_0_ represents the number of 0 values contained in each block, and *N* represents the number of 1 values contained in the block. The hash at all levels of the image can be calculated and generated by the following formula:

(10) $$\begin{array}{c} H_{1}=\left\{\begin{array}{cc} 0, & N_{0}\geq N_{1},\\ 1, & N_{0}<N_{1}. \end{array}\right) \end{array}$$

In the formula, 0 < *i* ≤ *M*. Moreover, each level of hash is composed of *M* bits. For a 512 × 512 image, using the above hash construction method, each level of features can generate a 40-bit hash code. The hash codes at all levels are scrambled, which can further enhance the security of the hash. Finally, all levels of hash are combined to generate the final perceptual hash code for authentication. The authentication hash with a code length of 120 bits can be generated for a 512 × 512 image.

It is not difficult to conclude from an examination of the perceptual hash authentication principle and current multiple perceptual authentication hash schemes that the security of the perceptual hash authentication algorithm is mostly determined by the security of the key in the scheme. The key to improving the security of the hash authentication algorithm is to improve the security of the key in the algorithm.

Aiming at the high-security key required by the perceptual hashing scheme, this paper proposes an optical key scheme based on the optical characteristics of the image.  Figure 4 is a schematic diagram of the generation of an optical key.

This paper takes optical distortion as an example to construct a key based on the optical characteristics of the image.

In optical distortion, the radial distortion model expressed in the image pixel coordinate system is generally written as

(11) $$\begin{array}{c} x_{d}=x_{c}+\left(x_{\mu }-x_{c}\right)\cdot T\left(r\right),\\ y_{d}=y_{c}+\left(y_{\mu }-y_{c}\right)\cdot T\left(r\right). \end{array}$$

Among them,

(12) $$\begin{array}{c} r=\sqrt{{\left(x_{\mu }-x_{c}\right)}^{2}{\left(y_{\mu }-y_{c}\right)}^{2}},\\ T\left(0\right)=1. \end{array}$$

In the formula, (*x*_*μ*_, *y*_*μ*_) are the coordinates of the ideal image point, (*x*_*d*_, *y*_*d*_) are the coordinates of the corresponding distorted image point, (*x*_*c*_, *y*_*c*_) are the coordinates of the distortion center, and *T*(·) is the distortion function.

If a polar coordinate system with the distortion center as the origin is used, the radial distortion model is simplified to *r*_*d*_=*r*_*μ*_ · *T*(*r*_*μ*_) and *T*(0)=1. Among them, *r*_*μ*_ is the radius coordinate of the ideal image point and *r*_*μ*_ is the radius coordinate of the corresponding distorted image point.

Then, the distortion function can be expressed as

(13) $$\begin{array}{c} T\left(r\right)=1+k_{1}r^{2}. \end{array}$$

The optical key generator *F* is defined as optical key *k*′ = *F* (key *k*, distortion parameter *k*_1_).

*F* is an optical key generation function that associates the key with the optical characteristics of the image itself, and XOR and other methods can be used to generate *F*. It can be seen that ordinary image signal processing (such as JPEG compression and filtering) will not affect the generated key. When the image is attacked by malicious tampering, it will cause the change of the hash key, which will seriously affect the generated hash code.

## 4. Analysis of the Effect of Intelligent Red Blood Cell Distribution Diagnosis Model on the Diagnosis and Treatment of Gastrointestinal Bleeding

The clinical data are 80 UGIH patients (UGIH group) admitted to our hospital from 2019 to December 2020, including 53 males and 27 females, aged 21–70 years. Admission criteria: all patients meet the diagnostic criteria for acute UGIH; the bleeding time of the patient is less than 24 hours; the patient has UGIH symptoms, such as melena or hematemesis, and coffee-like vomiting; the patient is accompanied by pale complexion, increased heart rate, and decreased blood pressure; the patient's vomit or stool routinely shows positive occult blood; the patient's liver and kidney functions are normal; and the patients do not have major bleeding after seeing a doctor. Exclusion criteria: patients have previous anaemia, blood system disease, tumor, liver and kidney disease, rheumatic disease, and so on, and patients have a recent history of surgery. In addition, 90 healthy patients are collected as a healthy control group.

Treatment method: symptomatic treatment is given to the UGIH group after admission. Moreover, the patient should take a lying position, keep the airway unobstructed, inhale oxygen if necessary, and fast during active bleeding. Simultaneously, vital signs must be carefully monitored, as well as the status of hematemesis and melena. In addition, aggressive blood volume supplementation and hemostasis treatments are required. After treatment, all patients recover and are discharged without death. The bleeding volume of the two groups of patients is counted, and the results obtained are shown in Table 1 and Figure 5.

On this basis, the recovery of the two groups of patients is analyzed, and the results obtained are shown in Table 2 and Figure 6.

With the increasing population of aging nationwide and the emergence of chronic noncommunicable diseases such as cardiovascular and cerebrovascular diseases, tumors, diabetes, and hypertension, UGIH has also become a common disease and is receiving increasing attention. UGIH refers to the gastrointestinal tract above the ligament of flexion, including bleeding caused by lesions such as esophagus, stomach, duodenum, pancreas, and gallbladder. It is a common clinical gastrointestinal emergency with complex causes and more dangerous conditions. In recent years, with the innovation and development of endoscopy technology, the diagnosis and treatment of UGIH patients have made great progress. RDW is a parameter that reflects the heterogeneity of red blood cell volume. It is measured by the coefficient of variation of red blood cell volume size, which is more objective and precise than examining red blood cells on blood smears for unequal morphological size. RDW may be used to diagnose iron deficiency anaemia and assess its effectiveness. The rise in RDW occurs before the reduction in MCV in iron-insufficiency anaemia, indicating early iron deficiency. When the MCV decreases, the RDW value increases more significantly. When the iron treatment is effective, the RDW will be larger than before the administration, and then it will gradually decrease to the normal level. In addition, UGIH is a common clinical emergency of the digestive tract, the disease is more dangerous, the pathogenesis is not clear, and domestic research on RDW in UGIH is still rare. Studying the role and value of RDW in UGIH will help expand the scope of UGIH research, open the situation that UGIH diagnosis is limited to existing technical means, and promote UGIH related research. At this stage, the gold standard for diagnosing UGIH is gastroscopy, but gastroscopy patients are more painful and mentally stressed. RDW can be measured in the patient's venous blood sample, which can reduce the patient's pain compared to gastroscopy. The introduction of RDW to study UGIH enriches UGIH diagnosis and treatment methods, provides more methods and parameters for clinical treatment of UGIH, and ensures the rapid and accurate diagnosis of UGIH.

Although medical technology has improved the clinical detection and treatment of upper gastrointestinal bleeding, some patients still experience rebleeding, which has a high death rate and a poor prognosis. The incidence of upper gastrointestinal bleeding accounts for 10%–20%, and rebleeding is an important predictor of death in patients with upper gastrointestinal bleeding. Most studies have shown that upper gastrointestinal bleeding is related to factors such as smoking, gender, heredity, and age.

RDW is a haematology analyzer-measured metric of the volume heterogeneity of surrounding red blood cells. It is a metric that measures the size difference between red blood cells. It is often used in conjunction with MCV for anaemia diagnosis and differentiation. Studies have found that high RDW is a poor prognostic sign of atherosclerosis, ischemic heart disease, acute and chronic heart failure, hypertension, and inflammatory bowel disease. Although the relationship between RDW and inflammation has not been fully elucidated, high RDW values are currently believed to be caused by chronic inflammation and malnutrition. Studies have found that inflammation and stress can cause red blood cell maturation disorders and affect the distribution width of red blood cells. The red blood cell distribution width index is positively correlated with inflammatory indicators such as IL-6 and TNF-*α*. Inflammatory factors may interfere with iron metabolism and affect bone marrow function, reducing the effect of erythropoietin and affecting the lifespan of red blood cells. Inflammatory factors can also inhibit the maturation of red blood cells and increase the number of abnormal red blood cells in the blood circulation, leading to an increase in RDW. In addition, inflammation can also change its morphology by changing ion channels and glycoproteins on the surface of the red blood cell membrane.

Red blood cell distribution width (RDW) is a parameter that the mountain blood analyzer measures to obtain the volume heterogeneity of the surrounding red blood cells. In short, it is an objective indicator that reflects the smallness of red blood cells because the red blood cell distribution width comes from proximity. Red blood cells detection data allow it to avoid the inaccuracy caused by man-made filmmaking elements and subjective impact when measuring red blood cell diameter and measure red blood cell diameter more directly. Objective and timely reflection of the unequal size of red blood cells is of great significance to the diagnosis and treatment of gastrointestinal bleeding.

## 5. Conclusion

RDW is a parameter of the volume heterogeneity of surrounding red blood cells measured by a haematology analyzer. It is an objective indicator reflecting the unequal size of red blood cells and is often used together with MCV for the diagnostic classification and differential diagnosis of anaemia. Studies have found that elevated RDW is a poor prognostic sign of atherosclerosis, ischemic heart disease, acute and chronic heart failure, hypertension, and inflammatory bowel disease. Although the relationship between RDW and inflammation has not been fully elucidated, high RDW values are currently believed to be caused by chronic inflammation and malnutrition. In addition, studies have found that inflammation and stress can cause red blood cell maturation disorders and affect the distribution of red blood cells. The red blood cell distribution width index is positively correlated with inflammatory indicators such as IL-6 and TNF-*α*. This paper studies the effect of red blood cell distribution width in the diagnosis of gastrointestinal bleeding based on this principle and validates the effect in combination with experiments. The red blood cell distribution width index may play an essential role in the diagnosis and management of gastrointestinal bleeding, according to the statistical findings.

## Figures and Tables

**Figure 1:** Block diagram of the realization process of the jitter quantization matrix.

**Figure 2:** Schematic diagram of extracting content-level features.

**Figure 3:** Schematic diagram of extracting features at all levels.

**Figure 4:** Schematic diagram of the optical key.

**Figure 5:** Line chart of gastrointestinal bleeding volume.

**Figure 6:** Line chart of the recovery situation of the test group and the control group.

**Table 1:** Comparison of gastrointestinal bleeding volume.

Number	Control group	Test group	Number	Control group	Test group
1	436.9	393.6	21	245.7	232.9
2	427.3	381.9	22	232.7	215.4
3	424.8	380.0	23	226.7	200.3
4	422.2	372.4	24	215.8	197.1
5	421.8	360.5	25	185.5	196.0
6	413.6	357.7	26	185.0	191.8
7	393.5	353.5	27	182.1	190.0
8	378.1	345.9	28	174.7	182.1
9	354.3	338.6	29	173.9	174.0
10	344.0	337.6	30	150.6	161.9
11	343.4	333.9	31	150.2	158.9
12	312.8	310.2	32	146.7	158.0
13	290.6	296.9	33	140.5	141.5
14	289.7	290.3	34	133.1	115.4
15	282.5	289.4	35	132.5	112.2
16	280.5	280.9	36	120.6	95.2
17	276.7	268.8	37	120.3	79.3
18	273.1	255.8	38	103.3	77.2
19	269.0	250.8	39	101.4	73.4
20	263.2	240.7	40	100.1	50.8

**Table 2:** Recovery situation of test group and control group.

Number	Control group	Test group	Number	Control group	Test group
1	95.8	89.4	21	83.3	93.5
2	89.4	91.9	22	88.4	94.5
3	82.9	94.8	23	74.6	92.2
4	94.4	93.1	24	84.6	89.9
5	82.5	93.6	25	84.9	89.4
6	72.8	96.8	26	85.4	92.6
7	93.6	91.1	27	85.3	95.5
8	74.0	96.0	28	78.8	95.5
9	87.4	92.2	29	75.8	91.2
10	84.8	91.8	30	72.6	96.9
11	78.6	92.8	31	82.4	92.4
12	80.1	92.6	32	78.0	92.5
13	96.8	95.5	33	87.5	89.3
14	84.6	93.7	34	75.1	92.5
15	88.6	89.4	35	90.4	89.6
16	77.0	92.6	36	83.6	92.1
17	94.7	92.2	37	96.3	96.1
18	89.4	93.9	38	86.4	93.2
19	94.5	94.6	39	72.2	94.8
20	74.9	91.3	40	92.8	92.1

## Data Availability

The data used to support the findings of this study are included within the article.

## References

[1] Lau J. Y. W., Yu Y., Tang R. S. Y. (2020). Timing of endoscopy for acute upper gastrointestinal bleeding. *New England Journal of Medicine*.

[2] Barkun A. N., Almadi M., Kuipers E. J. (2019). Management of n upper gastrointestinal bleeding: guideline recommendations from the international consensus group. *Annals of Internal Medicine*.

[3] Cook D., Guyatt G. (2018). Prophylaxis against upper gastrointestinal bleeding in hospitalized patients. *New England Journal of Medicine*.

[4] Oakland K., Chadwick G., East J. E. (2019). Diagnosis and management of acute lower gastrointestinal bleeding: guidelines from the British Society of Gastroenterology. *Gut*.

[5] Sung J. J., Chiu P. W., Chan F. K. L. (2018). Asia-Pacific working group consensus on non-variceal upper gastrointestinal bleeding: an update 2018. *Gut*.

[6] Kamboj A. K., Hoversten P., Leggett C. L. (2019). Upper gastrointestinal bleeding: e and management. *Mayo Clinic Proceedings*.

[7] Shung D. L., Au B., Taylor R. A. (2020). Validation of a machine learning model that outperforms clinical risk scoring systems for upper gastrointestinal bleeding. *Gastroenterology*.

[8] Wells M. L., Hansel S. L., Bruining D. H. (2018). CT for evaluation of acute gastrointestinal bleeding. *RadioGraphics*.

[9] Samuel R., Bilal M., Tayyem O., Guturu P. (2018). Evaluation and management of Non-variceal upper gastrointestinal bleeding. *Disease-a-Month*.

[10] Niikura R., Nagata N., Yamada A. (2020). Efficacy and safety of early vs elective colonoscopy for acute lower gastrointestinal bleeding. *Gastroenterology*.

[11] Gu Z.-C., Wei A.-H., Zhang C. (2020). Risk of major gastrointestinal bleeding with n conventional oral anticoagulants: a systematic review and meta-analysis. *Clinical Gastroenterology and Hepatology*.

[12] Miller C. S., Dorreen A., Martel M., Huynh T., Barkun A. N. (2017). Risk of gastrointestinal bleeding in patients taking non-vitamin K antagonist oral anticoagulants: a systematic review and meta-analysis. *Clinical Gastroenterology and Hepatology*.

[13] Chan F. K. L., Ching J. Y. L., Tse Y. K. (2017). Gastrointestinal safety of celecoxib versus naproxen in patients with cardiothrombotic diseases and arthritis after upper gastrointestinal bleeding (CONCERN): an industry-independent, double-blind, double-dummy, randomised trial. *The Lancet*.

[14] Chen W.-C., Lin K.-H., Huang Y.-T. (2017). The risk of lower gastrointestinal bleeding in low-dose aspirin users. *Alimentary Pharmacology & Therapeutics*.

[15] Cho S.-H., Lee Y.-S., Kim Y.-J. (2018). Outcomes and role of urgent endoscopy in high-risk patients with acute n gastrointestinal bleeding. *Clinical Gastroenterology and Hepatology*.

[16] Lanas-Gimeno A., Lanas A. (2017). Risk of gastrointestinal bleeding during anticoagulant treatment. *Expert Opinion on Drug Safety*.

[17] Converse M. P., Sobhanian M., Taber D. J., Houston B. A., Meadows H. B., Uber W. E. (2019). Effect of angiotensin II inhibitors on gastrointestinal bleeding in patients with left ventricular assist devices. *Journal of the American College of Cardiology*.

[18] Facciorusso A., Straus Takahashi M., Eyileten Postula C., Buccino V. R., Muscatiello N. (2019). Efficacy of hemostatic powders in upper gastrointestinal bleeding: a systematic review and meta-analysis. *Digestive and Liver Disease*.

[19] Kim J., Doyle J. B., Blackett J. W. (2020). Effect of the coronavirus 2019 pandemic on outcomes for patients admitted with gastrointestinal bleeding in New York city. *Gastroenterology*.

[20] Roberts I., Shakur-Still H., Afolabi A. (2020). Effects of a high-dose 24-h infusion of tranexamic acid on death and thromboembolic events in patients with acute gastrointestinal bleeding (HALT-IT): an international randomised, double-blind, placebo-controlled trial. *The Lancet*.

